The article "Postmenopausal women with osteoarthritis and osteoporosis show different ultrastructural characteristics of trabecular bone of the femoral head" was published in 2009. Journal: BMC Musculoskelet Disord.

# Postmenopausal women with osteoarthritis and osteoporosis show different ultrastructural characteristics of trabecular bone of the femoral head

**DOI:** 10.1186/1471-2474-10-35

**Published:** 2009-04-09

**Authors:** Yun Shen, Zi-Ming Zhang, Sheng-Dan Jiang, Lei-Sheng Jiang, Li-Yang Dai

**Affiliations:** 1 Department of Orthopaedic Surgery, Xinhua Hospital, Shanghai Jiaotong University School of Medicine, Shanghai, PR China

## Abstract

**Background:**

Osteoporosis (OP) and osteoarthritis (OA) are public health diseases affecting the quality of life of the elderly, and bring about a heavy burden to the society and family of patients. It has been debated whether or not there is an inverse relationship between these two disorders.

**Methods:**

To compare the exact difference in bone tissue structure between osteoporosis and osteoarthritis, we observed the ultrastructure of trabecular bone from the femoral heads using scanning electron microscopy (SEM) and transmission electron microscopy (TEM). A total of 15 femoral head specimens from postmenopausal women were collected during the procedures of total or hemi hip replacement (OP, n = 8; OA, n = 7). The morphologic structure of the trabecular bone, collagen fibers, resorption lacuna and osteoblasts were observed.

**Results:**

Under SEM, osteoporotic trabeculae appeared to be thinning, tapering, breaking and perforating. A number of resorption lacunae of various shapes were seen on the surface of the trabeculum. The collagen fibers of lacuna were resorbed. On occasion, naked granular bone crystals could be found. In the OA group, the trabecular bone looked thick with integrated structure. Reticular and granular new bone could be found. The trabeculum was covered by well-arranged collagen fibers around the resorption lacuna. In the OP group, under TEM, marginal collagen fibers were observed to be aligned loosely with enlarged spaces. A few inactive osteoblasts and no inflammatory cells were seen. In the OA group, the collagen fibers inside the trabeculum were arranged in a dense manner with many active osteoblasts and inflammatory cells infiltrating the matrix.

**Conclusion:**

We found significant differences in the trabecular bone, collagen fibers, lacunae and osteoblasts between postmenopausal women with OP and OA. These findings support the hypothesis that there is an inverse relationship between OP and OA.

## Background

Osteoporosis (OP) and osteoarthritis (OA) are two common diseases that severely influence quality of life, especially for the elderly. OP, characterized by the reduction in the amount of bone and deterioration of bone microarchitecture, is considered to be the consequence of an imbalance between bone formation and resorption. It also makes bone susceptible to fracture with increased bone fragility. OP is clinically defined as a condition in which bone mineral density (BMD) is at least 2.5 standard deviations (also referred to as 'T-score') below the mean of the young adult population by World Health Organization (WHO) [1]. OA is manifested by progressive degeneration of articular cartilage which is believed to be usually caused by articular cartilage erosion and chondrocyte damage [2]. The subchondral bone may play an important role in the pathogenesis of OA [3]. The sclerotic subchondral bone is considered to weaken the articular cartilage by impairing its ability to absorb mechanical shock, thereby influencing the progression of OA [4]. Although both OA and OP are strongly related to age and metabolism, they are multifaceted conditions influenced by mechanical and genetic factors [5-10].

Although the relationship between OA and OP remains controversial, an inverse relationship has been more widely accepted [11-14]. In clinical setting, both diseases rarely occurred in the same patient [15]. The femoral heads from osteoporotic fractures were found well preserved in earlier studies. Comparison of bone mineral densities (BMDs) in OA, OP and normal controls, the BMDs of osteoarthritic patients were the highest [16-19]. Even if patients with OA do suffer from osteoporotic fractures, the age at fracture occurrence is usually much older, which indicates that OA might have a protective effect on fracture [20].

The trabeculae in patients with OP have lower strength and are of poorer quality [21], whereas sclerotic subchondral trabecular bone is found in those with OA. However, the increase of stiffness in OA does not mean higher strength. Ding et al [22] reported that the thickness of trabeculae in early-staged OA patients increased significantly, but the strength of the subchondral trabecular bone was still weaker than healthy controls. Although the relationship between OA and OP has been investigated with regard to subchondral bone plates [23] or composition and mechanical properties of cancellous bone [4], the ultrastructure of trabecular bone has not been compared between these two diseases using both scanning electron microscopy (SEM) and transmission electron microscopy (TEM). An exploration of the ultrastructure of the trabecular bone, which contributes to the mechanical features, might be helpful to explain the real relationship between OA and OP populations. The aim of this study was to to investigate the trabecular ultrastructure between OA and OP using SEM and TEM with a working hypothesis for an inverse relationship between OA and OP.

## Methods

Femoral heads were obtained from 15 postmenopausal women with an average age of 76.8 (63–86 yrs) during hip replacement operations. Eight patients diagnosed with osteoporotic femoral neck fracture undertook a hemi-hip replacement, while the other seven with primary osteoarthritis sustained a total hip arthroplasty. To avoid disturbance of age and hormone level, each donor has at least five years menopause history. Each sample of articular cartilage from the OA group had severe erosion as defined by Outerbridge grade IV [24]. To ensure more consistent bone quality, patients with old osteoporotic fracture were precluded from this series. Any patients with osteomalacia, multiple myeloma, rheumatoid arthritis, or secondary osteoporosis due to hormone therapy were excluded from the OP group. Likewise, patients with congenital or acquired hip dysplasia, gout, rheumatoid arthritis or avascular necrosis of the femoral head were excluded from the OA group. The investigation was approved by institutional review board of our institution. In accordance with local ethical standards, informed consent was obtained from patients.

The femoral head was bivalved in the coronal plane with a sharp osteotome. The exposed surface was rinsed with saline solution repeatedly to remove blood and bone marrow. Then specimens, 5 mm × 5 mm × 5 mm in size for SEM and 2 mm × 2 mm × 2 mm for TEM, were harvested from the coronal medial plane from the trabecular structure of the femoral head, 1.5 cm below the joint surface [25,26]. All specimens were fixed with 2% glutaraldehyde solution, washed with 0.1 M sodium cacodylate buffer, and post-fixed with 1% osmium tetroxide. After dehydrating with an alcohol gradient series, different protocol was performed for SEM and TEM procedures. For SEM, after dehydrating with isoamyl acetate again, the specimen was dried using a critical point dryer with HCP-2. After being coated with a layer of gold, all specimens were studied under a scanning electron microscope (QUANTA-200, Philips, Eindhoven, The Netherlands). For TEM, each specimen was doubly replaced with propylene oxide, soaked with epoxy resin, and embedded in oven of 60°C for 48 hours. Specimens were then sectioned into ultra-thin slices, dyed with citric acid lead, and examined under a transmission electron microscope (CM-120, Philips, Eindhoven, The Netherlands).

## Results

### SEM

In the OP group, the cancellous bone of the femoral head was composed of either plate-like or rod-like trabeculae in the form of arch structures. However, the arch had been resorbed to become interrupted and form various stump structures. This phenomenon was more obvious in the rod-like trabeculae. Changes such as thinning, tapering, breakage, and perforation made the arch structure lose its integrity (Fig. 1A). The remaining trabeculae were short and sharp, like icicles. Some of them became round due to continuous resorption to obtain knob-like structure (Fig. 1B). These changes contributed to an obviously increasing separation of inter-trabeculae (Fig. 1C). Interestingly, the plate-like trabeculae maintained flat and broad structure integrated with rare breakage and perforation (Fig. 1D). Resorption of the trabecular bone occurred mainly at the central part of the arch structure. With progression of resorption, breakage and perforation took place (Fig. 2A).

**Figure 1:** **Images of trabecular bone in osteoporotic women under SEM**. A. Trabecular bone damaged due to resorptive activity. (×50). B. Icicle-like trabecular leave a stump structure after breakage. (×200). C. Large holes and cavities emerge between trabecular plates. (×100). D. Plate-like trabecular remain in a comparatively intact configuration. (×40).

**Figure 2:** **Images of trabecular bone head in osteoporotic women under SEM**. A. The middle part of trabecular bone was easy to penetrate and break as severe resorption activity occurred there. (×100). B. Resorption lacuna with paralleling collagen fibrils with broken fibrils on the bottom of it. (×3000). C. Newly generated collagen fibrils laying on the bottom of the lacuna in an ordered configuration. (×3000). D. Granular bone tissues with different heights surround the lacuna. (×3000).

Many resorption lacunae with oval, narrow oval or spindle shapes could be seen over the icicle-like trabeculae. The margin of the lacuna showed an irregular, perforated appearance. Adjacent lacunae were observed to have coalesced and fused together. Smooth and regular collagen fibrils could be discerned among the lacunae, namely on the unresorbed surface. Under high magnification, the collagen fibrils were of uniform size, existing in a parallel array orientation and showing oblique and finer connecting fibrils. Round, oval, or residual inorganic granules with irregular shape could be observed in the lacuna. On the bottom of the lacuna, tight or loose collagen fibrils presented irregular arrangement and breakage (Fig. 2B).

Resorption of the fibrils was also observed on the surface of the trabeculae among lacunae. Under high magnification, the collagen fibrils appeared loosely scattered and uneven, whereas the lacuna was shallow and empty with a perforated margin (Fig. 2C).

Between the spindle-shape resorption lacunae, the collagen fibril layer was incomplete and covered with needle-shape crystals. Vacant resorption lacunae mainly assembled near the lower position of the trabeculae. Under high magnification, uneven and irregular granules lacking specific orientation could be seen covering the space between the resorption lacunae. Occasionally, a few fibrils could be seen remaining at the bottom of the lacunae (Fig. 2D). These granules were arranged irregularly with a few thick collagen fibrils distributed irregularly (Fig. 3A).

**Figure 3:** **Images of trabecular bone in osteoporotic women under SEM. **A. few fibrils cross granular bone tissues obliquely. (×1200). B. Lacuna with elliptical shape. (×1500) C. New collagens lies on the bottom of the lacuna in an ordered configuration. (×3000).

Thinner collagen fibrils 0.5–1 μm in diameter and 5–10 μm in length, which represented the newly formed fibrils, emerged from inside the lacuna on the icicle-like trabecular bone (Fig. 3B). These fibrils appeared in a clear border arranged in a regular and parallel order. This origination extended from one side, filling up the bottom, towards the para-lacunar region on the opposite side (Fig. 3C).

In the OA group, the trabeculae of the femoral head maintained the intact arch structure, with bulky and bifurcate appearance (Fig. 4A). Under high magnification, the trabeculae were covered with regularly arranged collagen fibrils of similar orientation and diameter to form a cylindrical rather than an icicle-like network structure (Fig. 4B).

**Figure 4:** **Images of trabecular bone in osteoarthritic women under SEM**. A. Columned trabecular bone of the femoral head in women with OA. (×100). B. Formal collagen fibrils arrayed on the surface of the trabecuae. (×1500). C. Reticular new bone covering the trabeculae. (×3000). D. Some new bones merged. (×3000). E. Lacuna and orderly fibils on the bottom. (×3000). F. Granular new bone tissues inside the trabecular space. (×50).

The reticular new bone tissue formed by the thin fibril mesh could be found adhering to the surface of the trabeculae (Fig. 4C). Thicker fibers fused together to form a plate-like structure (Fig. 4D). A number of resorption lacunae generated by osteoclasts made the trabeculae a porous appearance. Thin and regular collagen fibrils were tightly arranged (Fig. 4E). A small amount of new bone formation was found in some lacunae with the occasional microfracture. Granular new bone appeared beside the reticular bone. The granular new bone gathered together with approximate size filling the space between the trabeculae (Fig. 4F). In comparison with the OP group, no inorganic bone crystal granules were present.

### TEM

In the OP group, some collagen fibers were found in regular arrays, while others appeared disorderly with almost no osteocytes observed, even under high magnification (Fig. 5A, 5B). Comparing the tight reticular structure with little space interior, the marginal collagen fibers were loose and irregular with large holes. Some of them fused together to different degrees to become large defects, just like a torn net (Fig. 5C). Osteoblasts with low activity scattered in the porous trabecular structure. The osteoblasts floating on the outer trabecular surface were elliptically shaped with protrusions that connected cells with each other (Fig. 5D, 6A). The nucleus was oval in fusiform cells. Some nuclei were large enough to match the width of the cell with little cytoplasm wrapping up. The big and irregular nucleolus varied in quantity in different osteoblasts. Some of them were darkly stained with more chromatins, whereas others were lightly stained (Fig. 6B). There were abundant ribosomes and vesicles scattered in the cytoplasm, but little rough endoplasmic reticulum and Golgi complex (Fig. 6C). Dying osteoblasts with irregular shape lost its own boundary, which made it difficult to identify the components of the cytoplasm. The vesicle increased while the mitochondrion and rough endoplasmic reticulum condensed (Fig. 6D). Although some osteoblasts were observed intact with regular appearance and rare protrusions, they were isolated from the bone surface (Fig. 6E). Under high magnification, chromatin was rarely found in these cells, while rough endoplasmic reticulum and Golgi complex were also scarce (Fig. 6F). No inflammatory cells were found in any osteoporotic specimen.

**Figure 5:** **Images of trabecular bone in osteoporotic women under TEM**. A, B. No osteocytes could be seen in the trabecular bone of femoral head in women with OP. (×3400) (×5800). C. Loose collagen fibrils on the edge of the trabecular bone. (×3400). D. Osteoblasts with depressed function floated on the surface of the bone. (Arrow points to the plasma of the osteoblast) (×7400).

**Figure 6:** **Images of trabecular bone and osteoblasts in osteoporotic women under TEM**. A. Strip-like plasma of osteoblast. (×7400). B. Spindly osteoblasts, some of which have double nucleoli. (×9700). C. Only a small quantity of rough endoplasmic reticulum and Glogi complex can be found. (×17500). D. One osteoblast was in the process of disaggregation. (×17500). E. Osteoblast above the trabecular bone. (×17500). F. Very little chromatin in the nucleolus. (×24000).

In OA group, the collagen fiber formed dense arrays with intercrossing fibers and appeared quite disorderly (Fig. 7A). Similar tight structures with little space also existed in outer surface of the trabeculae, unlike in the OP cases (Fig. 7B). Osteoblasts adhered to the bone surface, making the boundary unclear (Fig. 7C). Under high magnification, the large nucleus contributed to a high nucleus-cytoplasm ratio. The substance inside the cytoplasm was fairly condensed. Rough endoplasmic reticulum and Golgi complexes with active function were rich in the cytoplasm (Fig. 7D). In active area, osteoblasts with large and irregular nuclei were found distributed in clusters. Darkly stained nucleolus was due to abundant chromatins (Fig. 7E). Plenty of vesicles with different sizes were observed scattered among the rough endoplasmic reticulum which assembled in great pieces. Calcium salts were also shown in the interstitial substance (Fig. 7E, 7F). Under high magnification, rough endoplasmic reticulum arranged in orderly layers, while a few swollen mitochondria were also noted (Fig. 8A). Some osteoblasts had distinct boundaries while some did not. Osteoblasts connected with others by protrusions (Fig. 8B). New osteoblasts differentiated from osteogenic cells arrayed on the bone surface in columns to generate new bone (Fig. 8C). A few inflammatory cells could be found near the osteoblasts. They were elliptic or long-elliptic in shape with giant and sub-lobed nuclei which contained deep stained chromatins (Fig. 8D). They had no special location, sometimes outside the bone (Fig. 8D), while sometimes among the bone collagen fibers (Fig. 8E).

**Figure 7:** **Images of trabecular bone and osteoblasts in osteoarthritic women under TEM**. A. Trabecular bones in femoral heads of women with arthritis showed tightly arrayed structure with intercrossing fibrils. (×7400). B. No obvious space among the trabecular bones. (×3400). C. Part of osteoblasts integrated with trabecular bone. (×5800). D. One side of osteoblast integrated. (×7400). E. Vision field was full of osteoblasts. (×3400) F. Lots of rough endoplasmic reticulum and calcium salts in the osteoblasts. (×4200).

**Figure 8:** **Images of osteoblast and inflammatory cells in osteoarthritic women under TEM**. A. Rough endoplasmic reticulum with plenty of folds and swollen mitochondria. (×17500). B. Osteoblasts linked to the neighbouring one by prominence. (×7400). C. New columned osteoblasts in a ray. (×5800). D. Inflammatory cells. (×4200). E. One inflammatory cell infiltrated into the bone. (×4200).

## Discussion

Bone tissue is composed of two different components: organic and inorganic, which determine the toughness and rigidity, respectively. Both of these substances also serve the mechanical strength of the bone. Bone structure is composed of cortical and trabecular bone. While the former mainly bears mechanical load, the latter is more sensitive to hormones or other biological factors that are involved in modulating bone metabolism.

The mechanical properties of the trabecular bone are influenced by its microarchitechture, such as trabecular number, thickness, and spacing. Dilworth et al [27] noted significant difference in mean trabecular thickness between groups fed with or without zinc supplementation diets in an electron microscope study. The ratio of the trabecular nodes to terminations was considered as one of the important factors affecting bone strength. Other authors [28,29] also observed cortical bone under electron microscope.

Byers et al [30], who investigated more than 100 femoral heads excised from patients with femoral neck fracture, did not find any osteoarthritic change. In another epidemiological study in Jerusalem, the authors found that the incidence of OP and OA were 16.1% and 4.1%, respectively. However, only 0.5% had both diseases simultaneously [31]. Li et al [4] reported a trabecular bone loss of 17% in osteoporotic femoral heads, while a 60% increase was observed in patients with OA. The higher bone quantity and better mechanical quality could partly explain why femoral neck fractures were so rare in those people with OA [32]. However, Papadakis M et al [33] observed that the degree of lumbar lordosis was not associated with the presence of OA or OP. The reasons for the lack of difference may be due to, we believe, the size of sample, the criteria of subgroup, and the age of the patients.

In our present study, we found significant differences in the ultrastructure of the trabecular bone between OA and OP groups. Not only the structure but also collagen fibrils were shown intact in OA, whereas destructive changes were noted in OP. Meanwhile, more new bone formation could be observed in osteoarthritic donors. However, thinning and sparse trabecular bone was the most outstanding manifestation in the OP group. In addition, severe destructive changes in the rod-like trabeculae, such as sharpening and breakage, were shown in all specimens from the OP group. The similar appearance also occurred in the collagen fibrils on the trabecular surface to some extent. Any impairment in continuity and integrity might have a potential effect on bone strength. Results from TEM also supported that the increase in resorptive activity noted in OP patients might be related to more bone loss in comparison with OA. However, obviously increased new bone tissue in osteoarthritic samples implied that bone formation was more active than bone resorption. This finding is consistent with that reported by other authors [23]. As we know, most investigations by TEM focus on the cartilage or synovium of femoral head in OA. So the information about trabecular bone in OA under TEM was considerably limited.

The superficial layer of fibrils in OP varied in diameter, while some of them vanished to some degree. Similar changes were also observed in the deep layer fibrils. On the contrary, the collagen fibrils in both superficial and deep layers in OA remained intact and regular. Although this provides better bone toughness, more new bone tissue formation also increases bone stiffness, as described by the hypothesis proposed by Dequeker. [11]

Different kinds of new bone formation were observed in both OA and OP groups in this study. New collagen fibrils and bone matrix in the lacunae rarely existed in patients with OP, whereas reticular and granular new bone was shown widely in those with OA. Regularly arranged new collagen fibrils in the resorption lacunae implied that more active bone formation dominated bone turnover in osteoarthritic patients. However, those resorption lacunae also indicated high level of resorption in the OA group.

Collagen fibrils and matrix components could be synthesized and secreted by osteoblasts. In the present study, significant differences in appearance, number, and cellular organs of osteoblasts were shown between OA and OP groups. Osteoblasts in OP group demonstrated little function and scattered sparsely. Moreover, new osteoblasts were hardly seen in these osteoporotic donors. Conversely, a great number of osteoblasts with active function were noted in all specimens with OA. Thus, we suggested that more bone mass in OA population might be due to more active bone formation.

This study was limited by the nature of study as SEM and TEM is a 2-D method. By contrast, a micro-CT reconstruction is a powerful method to delineate structural characteristics of the trabecular bone in a 3-D fashion [34]. Therefore, a comparison between the OP and OA groups using 3-D micro-CT reconstruction would be necessary in the further studies.

Another limitation of this study might be the lack of quantitative data from electron microscopic findings. In fact, however, a 2-D histomorphometric analysis of cartilage and subchondral bone in postmenopausal women with OA and OP was made in our previous study [35]. In that study, lower bone volume fraction (BV/TV), trabecular thickness (Tb.Th), trabecular number (Tb.N) and the ratio of nodes to termini (Nd/Tm) were demonstrated in OP patients than OA patients, whereas increased trabecular space (Tb.Sp) was noted in these OP patients.

## Conclusion

In summary, we found significant differences in the ultrastructure of the trabecular bone between postmenopausal women with osteoporosis and osteoarthritis using SEM and TEM. These findings not only suggest totally different mechanism and progression of two common diseases, but also support the hypothesis that there is an inverse relationship between OA and OP. Bone resorption and formation activity of the trabecular bone prevail in OP and OA patients, respectively.

## Competing interests

The authors declare that they have no competing interests.

## Authors' contributions

All authors participated in the conception and design of the study. YS and ZMZ collected the data. All authors carried out data analysis and participated in the drafting of the manuscript.

## Pre-publication history

The pre-publication history for this paper can be accessed here:


